The article "Parameter Estimation in Step Stress Partially Accelerated Life Testing under Different Types of Censored Data" was published in 2022. Journal: Comput Intell Neurosci.

# Parameter Estimation in Step Stress Partially Accelerated Life Testing under Different Types of Censored Data

**DOI:** 10.1155/2022/3491732

**Published:** 2022-04-28

**Authors:** Mustafa Kamal, Sabir Ali Siddiqui, Ahmadur Rahman, Hassan Alsuhabi, Ibrahim Alkhairy, Thierno Souleymane Barry

**Affiliations:** ^1^Department of Basic Sciences, College of Science and Theoretical Studies, Saudi Electronic University, Dammam 32256, Saudi Arabia; ^2^Department of Mathematics and Sciences, College of Arts & Applied Sciences, Dhofar University, Salalah, Oman; ^3^Department of Statistics and Operations Research, Aligarh Muslim University, Aligarh, India; ^4^Department of Mathematics, Al-Qunfudah University College, Umm Al-Qura University, Mecca, Saudi Arabia; ^5^Mathematics (Statistics Option) Program, Pan African University Institute for Basic Sciences, Technology and Innovation (PAUSTI), 62000-00200 Nairobi, Kenya

## Abstract

A long testing period is usually required for the life testing of high-reliability products or materials. It is possible to shorten the testing process by using ALTs (accelerated life tests). Due to the fact that ALTs test products in harsher settings than are typical use conditions, the life expectancy of the objects they evaluate is reduced. Censored data in which the specific failure timings of all units assigned to test are not known, or all units assigned to test have not failed, may arise in ALTs for a variety of reasons, including operational failure, device malfunction, expense, and time restrictions. In this paper, we have considered the step stress partially accelerated life test (SSPALT) under two different censoring schemes, namely the type-I progressive hybrid censoring scheme (type-I PHCS) and the type-II progressive censorship scheme (type-II PCS). The failure times of the items are assumed to follow NH distribution, while the tampered random variable (TRV) model is used to explain the effect of stress change. In order to obtain the estimates of the unknown parameters, the maximum likelihood estimation (MLE) approach is adopted. Furthermore, based on the asymptotic theory of MLEs, the approximate confidence intervals (ACIs) are also constructed. The point estimates under two censoring schemes are compared in terms of root mean squared errors (RMSEs) and relative absolute biases (RABs), while ACIs are compared in terms of their lengths and coverage probabilities (CPs). The performance of the estimators has been evaluated and compared under two censoring schemes with various sample sizes through a simulation study. Simulation results show that estimates with type-I PHCS outperform estimates with type-II PCS in terms of RMSEs, RABs, lengths, and CPs. Finally, a real-world numerical example of insulating fluid failure times is presented to show how the approaches will work in reality.

The article "Parameter Estimation in Step Stress Partially Accelerated Life Testing under Different Types of Censored Data" was published in 2022. Journal: Comput Intell Neurosci.

## 1. Introduction

The customer's proclivity to place greater trust and happiness in a product has been thoroughly tested to ensure that it will fulfil its intended function with high reliability. Moreover, with the widespread use of computers, automation, and simulation, the overall quality of the manufacturing process has improved significantly, making the goods more reliable than their previous versions. Scientists require failure data to produce an efficient forecast about the product's expected life. Obtaining such failure data using ordinary life testing (OLT) is a time-consuming and expensive process for such highly reliable goods, and in such cases, OLTs are not suitable. As a solution, more sophisticated tests, such as ALTs and partial ALTs, are used to get rapid failures of goods by testing them under more severe conditions (such as temperature, voltage, humidity, and so on) than typical usage settings, resulting in decreased testing time, labor, and money.

In ALTs, products or materials are evaluated only at stress levels that are greater than the stress level at which they function in regular usage, with the hypothesis that a product's failure mechanisms and process will follow the same profile as when tested at normal stress. ALTs are often classified into three kinds depending on the stress loading modalities: constant stress ALT, step stress ALT, and progressive stress ALT (commonly abbreviated to CSALT, SSALT, and PSALT) [1, 2]. In CSALT, units are tested at more than one constant high stress level until all failures of all units are observed or the test is terminated for reasons such as a censoring scheme or an inexplicable failure cause. For further information, readers are directed to some good and relevant references, including [3–14] based on CSALT models. In SSALT, the testing units are initially subjected to a starting high level of stress; the failures are noted; and then the test items are removed at a prespecified time to test at the next level of stress, and so on. Many scholars have looked at the SSALT models, including [15–24]. PSALT, in which test units are exposed to gradually increasing stress over time to obtain failure data for testing, was initially proposed by [25]. In their study, they obtained estimates of the parameters of both the exponential and Weibull life distributions under PSALT. Ever since, numerous authors have looked at PSALT for various distributions and data kinds, including [26–30].

Censoring in life testing experiments can occur at any time, either intentionally or unintentionally. In intentional censoring, testing is ended after a specific period or a number of failures owing to cost and time limitations, whereas unintentional censoring is generally caused by operational failure or equipment malfunction. The most frequent types of intentional censoring are type-I (time-constrained) and type-II (failure-restricted). Because of the specified test termination time in type-I, an experiment may have a very low failure rate or even no failures, but the experiment length in type-II censoring may be rather long, rendering it impractical in many situations. Reference [31] proposed type-I hybrid censoring, which is basically a combination of type-I and type-II censoring, to circumvent these restrictions. One of the most significant shortcomings of type-I, type-II, and type-I hybrid censorings is that test items cannot be withdrawn at any time throughout the test other than the test termination points. More comprehensive censoring, such as type-II PCS and type-I PHCS, must be used in life testing studies to solve this issue [32]. In type-II PCS, a randomly selected sample of *n* items is first placed on an experiment with a predefined number of failures *m* and a preset randomized removing strategy *r*_1_, *r*_2_ …, *r*_*m*_. At the initial failure time *y*_1,*m*,*n*_, the experiment may proceed by removing *r*_1_ test items from the remaining *n* − 1 survivors. Similarly, at the second failure time *y*_2,*m*,*n*_, *r*_2_ test items will be removed from the remaining *n* − 1 − *r*_1_ survivals and so on until the *m*^*th*^ failure *y*_*m*,*m*,*n*_ occurs. When the *m*^*th*^ failure occurs, the test is stopped, and all the remaining *r*_*m*_=*n* − *m* − ∑_*i*=1_^*m*^*r*_*i*_ surviving survivors are eliminated. References [33–35] provide further details on type-II PCS. However, because of the preset size of observable failures, the major issue with type-II PCS is that the test length may be quite long, potentially resulting in additional expenditures and resources. Reference [36] introduces type-I PHCS with random terminal time *T*_0_^*∗*^=min(*y*_*m*,*m*,*n*_, *T*_0_) as a solution to this issue, where *T*_0_ is a preset test stoppage time. The most significant benefit of this censoring is that the test is now time-limited. See [32, 35, 36] for further details and insights.

The article "Parameter Estimation in Step Stress Partially Accelerated Life Testing under Different Types of Censored Data" was published in 2022. Journal: Comput Intell Neurosci.

In ALTs, the life of the test item at the stress level it will be used in real life is estimated by extrapolating the lifetime data obtained at high stress levels to the typical usage stress level. Although such life-stress links are very complicated or perhaps do not exist in some situations. To address this issue, PALTs, which may be thought of as a logical combination of OLTs and ALTs, are more suited for conducting life testing. In contrast to ALT, test units in PALT are allocated to both normal and accelerated circumstances in order to gather failure data. Furthermore, PALT does not require a life-stress relation to calculate the estimated life of a product under real-world conditions. CSPALT and SSPALT are two extensively utilized core PALT classifications. In CSPALT, product samples are tested under both regular and accelerated settings at the same time until the test is ended owing to a censoring scheme or an unforeseen malfunction. Readers can find more information about CSPALT models in [5, 37–40]. In SSPALT, products are tested up to prespecified time at normal use conditions, and then all products that still working are assigned to test on accelerated conditions until the test is ended owing to a censoring scheme or an unforeseen malfunction. To reflect the effect of stress change, [41] introduced the TRV model for SSPALT. More details on TRV models can be found in [41, 42].

Many studies for SSPALT based on different censoring schemes so far have been carried out; see [43–53] for example. Reference [47] considered the SSPALT based on the TRV model under type-II PCS to obtain the Bayes and ML estimates of the parameters of the Lomax distribution. Reference [48] estimated the parameters of the Weibull exponential distribution using the MLE approach based on SSPALT with type-II PCS. Reference [49] discussed the estimation of the stress-strength reliability under the assumption that the strength variable belongs to SSPALT and the components of strength and stress follow exponential distributions. Reference [50] described a *k*-stage SSPALT and derived model parameter estimates using interval type-I PCS with equal lengths of inspection interval. Reference [51] discussed and compared the MLEs of Weibull distribution parameters and AF based on adaptive type-I PHCS and type-I PHCS for SSPALT using the TRV model. Reference [52] investigated and compared MLEs of Burr type-XII distribution and AF under SSPALT based on the TRV model with type-I and adaptive type-II PHCS. Reference [53] produced parameter inferences based on SSPALT based on progressive hybrid censored masked data for a three-component hybrid system employing power-linear hazard rate distribution as lifetime distribution.

The NH distribution was proposed by [54] in 2011 as an extension of the exponential distribution. The NH distribution has some useful and appealing features, such as having an always zero mode and a closed-form HF that can explain increasing, decreasing, and constant hazard rates, making it an excellent choice in lifetime data analysis. As a specific case, particular probability distributions, such as the exponential distribution, may be generated. As a result, it is a feasible alternative to the Weibull, exponential, and gamma distributions. So far, several studies such as [55–63] considering the problem of estimation of the parameters of the NH distribution using MLE and BE techniques have been conducted. Assuming that the scale parameter of NH distribution has a log-linear relation with stress, [55] obtained MLEs of the parameters under CSALT and SSALT models. Under CSALT and PSALT for type-II PC data, [56, 57] considered the MLE and BE techniques to obtain the estimates of model parameters. Reference [59] explored optimum plans for *k*-level CSALT plans under complete data for NH distribution using D and C optimality. Recently, taking into account the MLE and BE techniques, [62] developed a CSPALT based on type-II PCS for estimating the parameters of the NH distribution. To the best of the authors' knowledge, there is no study based on SSPALT that discussed the estimation of the parameters of the NH distribution and the AF for type-II PCS and type-I PHCS. Reference [63] used the NH distribution as a lifetime distribution to estimate unknown model parameters in SSPALT with adaptive type-II PHCS and proposed two feasible optimum test approaches based on the A and D optimality.

The article "Parameter Estimation in Step Stress Partially Accelerated Life Testing under Different Types of Censored Data" was published in 2022. Journal: Comput Intell Neurosci.

This paper has two major goals: first, to present an SSPALT plan utilizing type-II PCS and type-I PHCS to estimate the parameters of the NH distribution and AF and, second, to compare the estimates using different sample combinations under the two mentioned censoring schemes. The remainder of the article is divided into the following sections: Section 2 discusses test assumptions and methodologies. In Section 3, SSPALT with type-II PCS is formulated, and MLEs and associated ACIs are produced. SSPALT with type-I PHCS is formulated and MLEs and associated ACIs are obtained in Section 4. In Section 5, for illustration purposes, a simulation study is carried out, and the results for the suggested models are discussed. In Section 6, a numerical example of insulating fluid failure times is utilized to show the applicability of the proposed estimation approach under SSPALT based on type-II PCS and type-I PHCS. Finally, Section 7 concludes the study with some remarks and future research directions.

## 2. Test Assumptions and Procedure

In this article, for both type II-PCS and type I-PHCS data, we made the following assumptions under SSPALT:

a1: The SSPALT is formulated using two stress levels *S*_*u*_ and *S*_*a*_(*S*_*u*_ < *S*_*a*_), where *S*_*u*_ represents use (normal) stress conditions and *S*_*a*_ represents severe (accelerated) stress conditions.
a2: There are *n* items that are put on the life test, which are identical and independent in nature. At least one failure at each stress *S*_*u*_ and *S*_*a*_ must be observed.
a3: The failure time *T* of each test item follows the NH distribution, with the probability density function (PDF), cumulative distribution function (CDF), survival function (SF), and hazard rate function (HRF) provided by
  (1) $$\begin{array}{c} f\left(t;\alpha ,\theta \right)=\alpha \theta {\left(1+\theta t\right)}^{\alpha -1}\text{exp}\left[1-{\left(1+\theta t\right)}^{\alpha }\right],t>0,\alpha >0,\theta >0, \end{array}$$
  (2) $$\begin{array}{c} F\left(t;\alpha ,\theta \right)=1-\text{exp}\left[1-{\left(1+\theta t\right)}^{\alpha }\right],t>0,\alpha >0,\theta >0, \end{array}$$
  (3) $$\begin{array}{c} R\left(t\right)=\text{exp}\left[1-{\left(1+\theta t\right)}^{\alpha }\right],t>0,\alpha >0,\theta >0, \end{array}$$
  (4) $$\begin{array}{c} h\left(t\right)=\alpha \theta {\left(1+\theta t\right)}^{\alpha -1},t>0,\alpha >0,\theta >0, \end{array}$$
where *θ* and *α* represents the scale and shape parameters of the distribution, respectively.  Figure 1 displays various shapes of PDF and HRF generated with varying input values of parameters.
a4: All *n* units are initially tested under stress *S*_*u*_ until a prespecified stress change time *τ*, at which point all surviving survivors are moved to be tested at stress *S*_*a*_. The switching impact of stress on product life from *S*_*u*_ to *S*_*a*_ can be determined by multiplying inverse of AF by the residual life of the product, and total life *Y* at *S*_*a*_ may theoretically be described by the TRV model as follows:
  (5) $$\begin{array}{c} Y=\left\{\begin{array}{c} T\text{if}T\leq \tau \\ \tau +\beta^{-1}\left(T-\tau \right)\text{if}T>\tau , \end{array}\right) \end{array}$$
where *T* is the lifespan of the test unit at condition *S*_*u*_ and *β* > 1 is the AF, which is in general depends on the *S*_*u*_ and *S*_*a*_. Now, we can describe the PDF and RF of *Y* based on a4 as follows:
  (6) $$\begin{array}{c} f\left(y\right)=\left\{\begin{array}{c} 0\text{if}y\leq 0,\\ f_{1}\left(y\right)\text{if}0<y\leq \tau ,\\ f_{2}\left(y\right)\text{if}y>\tau , \end{array}\right) \end{array}$$
  (7) $$\begin{array}{c} R\left(y\right)=\left\{\begin{array}{c} 0\text{if}y\leq 0,\\ R_{1}\left(y\right)\text{if}0<y\leq \tau ,\\ R_{2}\left(y\right)\text{if}y>\tau . \end{array}\right) \end{array}$$

Using equations (1), (2), (5)–(7), the following expressions can be obtained easily:

(8) $$\begin{array}{c} f\left(y\right)=\left\{\begin{array}{c} 0\text{if}y\leq 0,\\ f_{1}\left(y;\alpha ,\theta \right)=\alpha \theta {\left(1+\theta y\right)}^{\alpha -1}\text{exp}\left[1-{\left(1+\theta y\right)}^{\alpha }\right]\text{if}0<y\leq \tau ,\\ f_{2}\left(y\right)=\alpha \beta \theta {\left[1+\theta \left(\tau +\beta \left(y-\tau \right)\right)\right]}^{\alpha -1}\text{exp}\left[1-{\left\{1+\theta \left(\tau +\beta \left(y-\tau \right)\right)\right\}}^{\alpha }\right]\text{if}y>\tau , \end{array}\right) \end{array}$$

(9) $$\begin{array}{c} R\left(y\right)=\left\{\begin{array}{c} 0\text{if}y\leq 0,\\ R_{1}\left(y;\alpha ,\theta \right)=\text{exp}\left[1-{\left(1+\theta y\right)}^{\alpha }\right]\text{if}0<y\leq \tau ,\\ R_{2}\left(y\right)=\text{exp}\left[1-{\left\{1+\theta \left(\tau +\beta \left(y-\tau \right)\right)\right\}}^{\alpha }\right]\text{if}y>\tau . \end{array}\right) \end{array}$$

The article "Parameter Estimation in Step Stress Partially Accelerated Life Testing under Different Types of Censored Data" was published in 2022. Journal: Comput Intell Neurosci.

## 3. SSPALT Formulation and Parameter Inference with Type-II PCS

In this section, we determined the MLEs and ACIs of the parameters using the SSPALT model and type-II PCS. Assume that all *n* components/items are assigned to stress level *S*_*u*_ to begin the testing process with some of the prespecified test restrictions *τ*, *m*, and *r*_1_, *r*_2_ …, *r*_*m*_(*τ* <  *m* < *n*). Continue the experiment at stress *S*_*u*_ until time *τ*, assuming that *y*_1,*m*,*n*_ < *y*_2,*m*,*n*_ < ⋯<*y*_*n*_1_,*m*,*n*_ are the failure data observed before *τ* and *r*_1_, *r*_2_ …, *r*_*n*_1__ are the total number of items eliminated at usage stress *S*_*u*_ due to the type-II PCS. All components/items that have not failed/been removed by time *τ* are now allocated to test at *S*_*a*_, and the experiment continues to run in the same manner as at *S*_*u*_ until the occurrence of *m*^th^ failure. The observed failure sample at *S*_*a*_ is *y*_*n*_1_+1,*m*,*n*_ < *y*_*n*_1_+2,*m*,*n*_ < ⋯<*y*_*m*,*m*,*n*_, and the total removals are *r*_*n*_1_+1_, *r*_*n*_1_+2_ …, *r*_*n*_1_+*m*_. Finally, when *m*^*th*^ failure is observed, the test is stopped, and all remaining *r*_*m*_=*n* − *m* − ∑_*i*=1_^*m*−1^*r*_*i*_ test items that have not yet failed are removed from the experiment.

The test description makes it clear that the total number of failures observed at *S*_*u*_ prior to time *τ* is *n*_1_, and consequently, (*m* − *n*_1_) is the total number of failures observed at *S*_*a*_. Under SSPALT, the entire observed failure data with type-II PCS of size *m* will now be of the form *y*_1,*m*,*n*_ < *y*_2,*m*,*n*_ < ⋯<*y*_*n*_1_,*m*,*n*_ ≤ *τ* < *y*_*n*_1_+1,*m*,*n*_ < ⋯<*y*_*m*,*m*,*n*_, and therefore, the appropriate likelihood function may thus be expressed as follows:

(10) $$\begin{array}{c} L\left(y,\;\alpha ,\;\theta ,\;\beta \right)=C\prod_{i=1}^{n_{1}}f_{1}\left(y_{i}\right){\left[R_{1}\left(y_{i}\right)\right]}^{r_{i}}\;\prod_{i=n_{1}+1}^{m}f_{2}\left(y_{i}\right){\left[R_{2}\left(y_{i}\right)\right]}^{r_{i}}, \end{array}$$

where *C*=*n* (*n* − 1 − *r*_1_)(*n* − 2 − *r*_1_ − *r*_2_) … (*n* − *m*)(*n* − *m* − ∑_*i*=1_^*m*−1^*r*_*i*_) and *y*_*i*_=*y*_*i*,*m*,*n*_, *i*=1,2,3 … *m*. Now using equations (1), (3), (8), and (9), and equation (10) can be rewritten as follows:

(11) $$\begin{array}{c} L\left(y,\alpha ,\theta ,\beta \right)=C\overset{n_{1}}{\underset{i=1}{\prod }}\alpha \theta {\left(A\left(y_{i}\right)\right)}^{\alpha -1}\text{exp}\left\{1-{\left(A\left(y_{i}\right)\right)}^{\alpha }\right\}{\left\{\text{exp}\left[1-{\left(A\left(y_{i}\right)\right)}^{\alpha }\right]\right\}}^{r_{i}}\;\\ \prod_{i=n_{1}+1}^{m}\alpha \beta \theta {\left\{B\left(y_{i}\right)\right\}}^{\alpha -1}\text{exp}\left\{1-{\left(B\left(y_{i}\right)\right)}^{\alpha }\right\}{\left\{\text{exp}\left[1-{\left(B\left(y_{i}\right)\right)}^{\alpha }\right]\right\}}^{r_{i}}, \end{array}$$

where *A*(*y*_*i*_)=(1+*θy*_*i*_), *B*(*y*_*i*_)={1+*θ*(*τ*+*β*(*y*_*i*_ − *τ*))}, and *B*(*y*_*i*_) − 1=*θ*(*τ*+*β*(*y*_*i*_ − *τ*)). Now, the log-likelihood Log(*y*, *α*, *θ*, *β*)=*ℓ* of equation (11) can be derived as follows:

(12) $$\begin{array}{c} \ell =\text{log}C+m\text{log}\alpha +m\text{log}\theta +\left(m-n_{1}\right)\text{log}\beta +\left(\alpha -1\right)\overset{n_{1}}{\underset{i=1}{\sum }}\log\left(A\left(y_{i}\right)\right)-\overset{n_{1}}{\underset{i=1}{\sum }}\left(r_{i}+1\right){\left(A\left(y_{i}\right)\right)}^{\alpha }+\left(\alpha -1\right)\overset{m}{\underset{i=n_{1}+1}{\sum }}\text{log}\left[B\left(y_{i}\right)\right]-\overset{m}{\underset{i=n_{1}+1}{\sum }}\left(r_{i}+1\right){\left[B\left(y_{i}\right)\right]}^{\alpha }. \end{array}$$

The article "Parameter Estimation in Step Stress Partially Accelerated Life Testing under Different Types of Censored Data" was published in 2022. Journal: Comput Intell Neurosci.

### 3.1. Point Estimates

Now, by differentiating (12) with respect to *α*, *β*and*θ*, the following equations are obtained:

(13) $$\begin{array}{c} \frac{\partial \ell }{\partial \alpha }=\frac{m}{\alpha }+\overset{n_{1}}{\underset{i=1}{\sum }}\log\left(A\left(y_{i}\right)\right)-\alpha \overset{n_{1}}{\underset{i=1}{\sum }}\left(1+r_{i}\right){\left(A\left(y_{i}\right)\right)}^{\alpha }\log\left(A\left(y_{i}\right)\right)+\overset{m}{\underset{i=n_{1}+1}{\sum }}\text{log}\left\{B\left(y_{i}\right)\right\}-\overset{n_{1}+n_{2}}{\underset{i=n_{1}+1}{\sum }}\left(1+r_{i}\right){\left\{B\left(y_{i}\right)\right\}}^{\alpha }\text{log}\left\{B\left(y_{i}\right)\right\}=0, \end{array}$$

(14) $$\begin{array}{c} \frac{\partial \ell }{\partial \beta }=\frac{\left(m-n_{1}\right)}{\beta }+\left(\alpha -1\right)\theta \overset{m}{\underset{i=n_{1}+1}{\sum }}\frac{\left(y_{i}-\tau \right)}{\left\{B\left(y_{i}\right)\right\}}-\alpha \theta \overset{m}{\underset{i=n_{1}+1}{\sum }}\left(1+r_{i}\right)\left(y_{i}-\tau \right){\left\{B\left(y_{i}\right)\right\}}^{\alpha -1}=0, \end{array}$$

(15) $$\begin{array}{c} \frac{\partial \ell }{\partial \theta }=\frac{m}{\theta }+\left(\alpha -1\right)\overset{n_{1}}{\underset{i=1}{\sum }}\frac{y_{i}}{\left(A\left(y_{i}\right)\right)}-\alpha \overset{n_{1}}{\underset{i=1}{\sum }}\left(1+r_{i}\right){\left(A\left(y_{i}\right)\right)}^{\alpha -1}+\left(\alpha -1\right)\overset{m}{\underset{i=n_{1}+1}{\sum }}\frac{\tau +\beta \left(y_{i}-\tau \right)}{\left\{B\left(y_{i}\right)\right\}}-\alpha \overset{m}{\underset{i=n_{1}+1}{\sum }}\left(1+r_{i}\right)\left(\tau +\beta \left(y_{i}-\tau \right)\right){\left\{B\left(y_{i}\right)\right\}}^{\alpha -1}=0. \end{array}$$

The MLEs $\left(\hat{\alpha },\hat{\theta },\hat{\beta }\;\right)$ of the unknown parameters (*α*, *θ*, *β*) of the model discussed here can be obtained by solving equations (13)–(15) simultaneously. Unfortunately, the system of equations (13)–(15) is nonlinear; therefore, no closed-form solution can be obtained analytically. As a result of this problem, some iterative methods must be used to obtain estimates of unknown parameters (*α*, *θ*, *β*) of the model. There are several iterative approaches, such as the Newton–Raphson method for solving nonlinear equations. In this case, we implemented the optim () function of the R statistical software/language to solve our nonlinear equations.

### 3.2. Interval Estimates

In this subsection, using the asymptotic properties of MLEs, we determine the ACIs of model parameters. Given specific regularity requirements, asymptotic features indicate that MLEs are approximately distributed according to the normal distribution with mean zero and variance (*F*)^−1^, which can be represented mathematically as follows:

(16) $$\begin{array}{c} \left(\hat{\alpha }-\alpha ,\hat{\theta }-\theta ,\hat{\beta }-\beta \right)∼N\left(0,{\left(F\right)}^{-1}\;\right), \end{array}$$

where (*F*)^−1^ is the inverse of the observed Fisher information matrix and is commonly referred to as a variance-covariance matrix for MLEs. It is possible to derive it as follows:

(17) $$\begin{array}{c} {\left(F\right)}^{-1}={\left[-\begin{array}{ccc} -\frac{\partial^{2}\ell }{\partial \alpha^{2}} & -\frac{\partial^{2}\ell }{\partial \alpha \;\partial \theta } & -\frac{\partial^{2}\ell }{\partial \alpha \;\partial \beta }\\ \frac{\partial^{2}\ell }{\partial \theta \;\partial \alpha } & -\frac{\partial^{2}\ell }{\partial \theta^{2}} & -\frac{\partial^{2}\ell }{\partial \beta \;\partial \theta }\\ -\frac{\partial^{2}\ell }{\partial \beta \;\partial \alpha } & -\frac{\partial^{2}\ell }{\partial \theta \;\partial \beta } & -\frac{\partial^{2}\ell }{\partial \beta^{2}} \end{array}\right]}_{\left(\hat{\alpha },\hat{\theta },\hat{\beta }\right)}^{-1}=\left[\begin{array}{ccc} \text{var}\left(\hat{\alpha }\right) & \text{covar}\left(\hat{\alpha }\theta \right) & \text{covar}\left(\hat{\alpha }\hat{\beta }\right)\\ \text{covar}\left(\hat{\theta }\hat{\alpha }\right) & \text{var}\left(\hat{\theta }\right) & \text{covar}\left(\hat{\beta }\hat{\theta }\right)\\ \text{covar}\left(\hat{\beta }\hat{\alpha }\right) & \text{covar}\left(\hat{\theta }\hat{\beta }\right) & \text{var}\left(\hat{\beta }\right) \end{array}\right]. \end{array}$$

The elements of *F* can be expressed by the following equations:

(18) $$\begin{array}{c} \frac{\partial^{2}\ell }{\partial \alpha^{2}}=-\frac{m}{\alpha^{2}}-\overset{n_{1}}{\underset{i=1}{\sum }}\left(1+r_{i}\right){\left(A\left(y_{i}\right)\right)}^{\alpha }{\left\{\log\left(A\left(y_{i}\right)\right)\right\}}^{2}-\overset{m}{\underset{i=n_{1}+1}{\sum }}\left(1+r_{i}\right){\left\{B\left(y_{i}\right)\right\}}^{\alpha }{\left\{\text{log}\left[B\left(y_{i}\right)\right]\right\}}^{2}\\ \frac{\partial^{2}\ell }{\partial \theta^{2}}=-\frac{m}{\theta^{2}}-\left(\alpha -1\right)\overset{n_{1}}{\underset{i=1}{\sum }}\frac{y_{i}{}^{2}}{{\left(A\left(y_{i}\right)\right)}^{2}}-\alpha \left(\alpha -1\right)\overset{n_{1}}{\underset{i=1}{\sum }}\left(1+r_{i}\right)y_{i}{}^{2}{\left(A\left(y_{i}\right)\right)}^{\alpha -2}\\ -\left(\alpha -1\right)\overset{m}{\underset{i=n_{1}+1}{\sum }}\frac{{\left(\tau +\beta \left(y_{i}-\tau \right)\right)}^{2}}{{\left\{B\left(y_{i}\right)\right\}}^{2}}-\alpha \left(\alpha -1\right)\overset{m}{\underset{i=n_{1}+1}{\sum }}\left(1+r_{i}\right){\left(\tau +\beta \left(y_{i}-\tau \right)\right)}^{2}{\left\{B\left(y_{i}\right)\right\}}^{\alpha -2}\\ \frac{\partial^{2}\ell }{\partial \beta^{2}}=-\frac{\left(m-n_{1}\right)}{\beta^{2}}-\left(\alpha -1\right)\theta^{2}\overset{m}{\underset{i=n_{1}+1}{\sum }}\frac{{\left(y_{i}-\tau \right)}^{2}}{{\left\{B\left(y_{i}\right)\right\}}^{2}}-\alpha \left(\alpha -1\right)\theta^{2}\overset{m}{\underset{i=n_{1}+1}{\sum }}\left(1+r_{i}\right){\left(y_{i}-\tau \right)}^{2}{\left\{B\left(y_{i}\right)\right\}}^{\alpha -2}\\ \frac{\partial^{2}\ell }{\partial \theta \;\partial \alpha }=\frac{\partial^{2}\ell }{\partial \alpha \;\partial \theta }=\overset{n_{1}}{\underset{i=1}{\sum }}\frac{y_{i}}{\left(A\left(y_{i}\right)\right)}-\overset{n_{1}}{\underset{i=1}{\sum }}\left(1+r_{i}\right)y_{i}{\left(A\left(y_{i}\right)\right)}^{\alpha -1}\left\{1+\alpha \text{ log}\left(A\left(y_{i}\right)\right)\right\}+\overset{m}{\underset{i=n_{1}+1}{\sum }}\frac{\tau +\beta \left(y_{i}-\tau \right)}{\left\{B\left(y_{i}\right)\right\}}-\overset{m}{\underset{i=n_{1}+1}{\sum }}\left(1+r_{i}\right)\left(\tau +\beta \left(y_{i}-\tau \right)\right){\left\{B\left(y_{i}\right)\right\}}^{\alpha -1}\left\{1+\alpha \text{ log}\left[B\left(y_{i}\right)\right]\right\}\\ \frac{\partial^{2}\ell }{\partial \alpha \;\partial \beta }=\frac{\partial^{2}\ell }{\partial \beta \;\partial \alpha }=\theta \overset{m}{\underset{i=n_{1}+1}{\sum }}\frac{\left(y_{i}-\tau \right)}{\left\{B\left(y_{i}\right)\right\}}-\overset{m}{\underset{i=n_{1}+1}{\sum }}\left(1+r_{i}\right)\left(y_{i}-\tau \right){\left\{B\left(y_{i}\right)\right\}}^{\alpha -1}\left\{1+\alpha \text{ log}\left[B\left(y_{i}\right)\right]\right\}\\ \frac{\partial^{2}\ell }{\partial \theta \;\partial \beta }=\frac{\partial^{2}\ell }{\partial \beta \;\partial \theta }=\left(\alpha -1\right)\overset{n_{1}+n_{2}}{\underset{i=n_{1}+1}{\sum }}\frac{\left(y_{i}-\tau \right)}{{\left\{B\left(y_{i}\right)\right\}}^{2}}+\alpha \overset{n_{1}+n_{2}}{\underset{i=n_{1}+1}{\sum }}\left(1+r_{i}\right)\left(y_{i}-\tau \right){\left\{B\left(y_{i}\right)\right\}}^{\alpha -2}\left\{B\left(y_{i}\right)\right\}. \end{array}$$

Now, two-sided 100(1 − Δ)% ACIs for the parameter *α*, *θ*, and *β* can be obtained as follows:

(19) $$\begin{array}{c} \hat{\alpha }\pm Z_{\Delta /2}\sqrt{\mathrm{var}\left(\hat{\alpha }\right)};\hat{\theta }\pm Z_{\Delta /2}\sqrt{\mathrm{var}\left(\hat{\theta }\right)};\hat{\beta }\pm Z_{\Delta /2}\sqrt{\mathrm{var}\left(\hat{\beta }\right)}, \end{array}$$

where ±*Z*_Δ/2_ represents standard normal distribution's upper and lower Δ/2^th^ percentile. $\mathrm{var}\left(\hat{\alpha }\right),\mathrm{var}\left(\hat{\theta }\right)$, and $\mathrm{var}\left(\hat{\beta }\right)$ are the diagonal entries of (*F*)^−1^.

The article "Parameter Estimation in Step Stress Partially Accelerated Life Testing under Different Types of Censored Data" was published in 2022. Journal: Comput Intell Neurosci.

## 4. SSPALT Formulation and Parameter Inference with Type-I PHCS

In this section, SSPALT with type-I PHCS will be formulated first, followed by MLEs and ACIs of model parameters. In SSPALT with type-I PHCS, a random sample of *n* test items is randomly allocated for testing under stress *S*_*u*_ with prefixed experimental restrictions *τ*, *m*, *T*_0_ and progressive removal pattern *r*_1_, *r*_2_ …, *r*_*m*_. Now, *r*_*i*_, *i*=1,2,   … *n*_1_ test items are removed from the test randomly at *i*^*th*^ failure observation *y*_*i*,*m*,*n*_ and the experiment continue to run until time *τ*(*τ* ≥ *y*_*n*_1__). At time *τ*, all of the survivors *n* − *n*_1_ − ∑_*i*=1_^*n*_1_−1^*r*_*i*_ at *S*_*u*_ are removed and then assigned for testing at *S*_*a*_ until the random termination time *T*_0_^*∗*^=min(*y*_*m*,*m*,*n*_, *T*_0_) of the experiment. For *y*_*m*,*m*,*n*_ ≤ *T*_0_, this means that the *m*^*th*^ failure *y*_*m*,*m*,*n*_ is observed before time *T*_0_, and the test is stopped at *m*^*th*^ failure time *y*_*m*,*m*,*n*_ by removing all the remaining survivals *r*_*m*_=*n* − *m* − ∑_*i*=1_^*m*−1^*r*_*i*_. For *y*_*m*,*m*,*n*_ > *T*_0_, this means *m*^*th*^ failure is not observed before time *T*_0_, and only *J* failures are observed; then, at time *T*_0_, test will be terminated by removing all *r*_*m*_=*n* − *J* − ∑_*i*=1_^*J*^*r*_*i*_ remaining survivals. Hence, under SSPALT with type-I PHCS, we observed two types of data: (i) *y*_1,*m*,*n*_ < *y*_2,*m*,*n*_ < ⋯<*y*_*n*_1_,*m*,*n*_ ≤ *τ* < *y*_*n*_1_+1,*m*,*n*_ < ⋯<*y*_*m*,*m*,*n*_if*y*_*m*,*m*,*n*_ ≤ *T*_0_ and (ii) *y*_1,*m*,*n*_ < *y*_2,*m*,*n*_ < ⋯<*y*_*n*_1_+1,*m*,*n*_ ≤ *τ* < *y*_*n*_1_+1,*m*,*n*_ < ⋯<*y*_*J*,*m*,*n*_if*y*_*J*,*m*,*n*_ ≤ *T*_0_ < *y*_*n*_1_+*n*_2_,*m*,*n*_.

Suppose that *n*_1_ is the size of failure sample observed at *S*_*u*_ before time *τ* and *n*_2_ is the size of the observed failure sample at *S*_*a*_ after time *τ*. Under SSPALT, the entire observed failure data with type-type-I PHCS will now be of the form *y*_1,*m*,*n*_ < *y*_2,*m*,*n*_ < ⋯<*y*_*n*_1_,*m*,*n*_ ≤ *τ* < *y*_*n*_1_+1,*m*,*n*_ < ⋯<*y*_*m*,*m*,*n*_ ≤ *T*_0_, and therefore, the appropriate likelihood function may be expressed as follows:

(20) $$\begin{array}{c} L\left(y,\alpha ,\theta ,\beta \right)=C\prod_{i=1}^{n_{1}}f_{1}\left(y_{i}\right){\left[R_{1}\left(y_{i}\right)\right]}^{r_{i}}\prod_{i=n_{1}+1}^{n_{1}+n_{2}}f_{2}\left(y_{i}\right)\;{\left[R_{2}\left(y_{i}\right)\right]}^{r_{i}}{\left[R_{2}\left(T_{0}\right)\right]}^{r}, \end{array}$$

where *C*=*n* (*n* − 1 − *r*_1_)(*n* − 2 − *r*_1_ − *r*_2_) ⋯ (*n* − *J* − ∑_*i*=1_^*m*−1^*r*_*i*_); for case (i), *n*_1_+*n*_2_=*m*; and for case (ii), *n*_1_+*n*_2_=*J*. *y*_*n*_1_+*j*,*m*,*n*_,…, *y*_*m*,*m*,*n*_ are not observed. Now using equations (1), (3), (8), (9), and (23) can be rewritten as follows:

(21) $$\begin{array}{c} L\left(y,\;\alpha ,\;\theta ,\;\beta \right)=C{\prod_{i=1}^{n_{1}}\alpha \theta \left(A\left(y_{i}\right)\right)}^{\alpha -1}\text{exp}\left\{1-{\left(A\left(y_{i}\right)\right)}^{\alpha }\right\}{\left[\text{exp}\left\{1-{\left(A\left(y_{i}\right)\right)}^{\alpha }\right\}\right]}^{r_{i}}\\ {\prod_{i=n_{1}+1}^{n_{1}+n_{2}}\alpha \beta \theta \left\{B\left(y_{i}\right)\right\}}^{\alpha -1}\text{exp}\left\{1-{\left(B\left(y_{i}\right)\right)}^{\alpha }\right\}{\left[\text{exp}\left\{1-{\left(B\left(y_{i}\right)\right)}^{\alpha }\right\}\right]}^{r_{i}}{\left[\text{exp}\left\{1-{\left(B\left(T_{0}\right)\right)}^{\alpha }\right\}\right]}^{r}, \end{array}$$

where *A*(*y*_*i*_)=(1+*θy*_*i*_), *B*(*y*_*i*_)={1+*θ*(*τ*+*β*(*y*_*i*_ − *τ*))}, and *B*(*T*_0_)={1+*θ*(*τ*+*β*(*T*_0_ − *τ*))}. Now, log-likelihood Log(*y*, *α*, *θ*, *β*)=*l* of equation (24) can be derived as follows:

(22) $$\begin{array}{c} l=\text{log}C+\left(n_{1}+n_{2}\right)\left(\text{log}\alpha +\text{log}\theta \right)+n_{2}\text{log}\beta +n_{2}r\left\{1-{\left(B\left(T_{0}\right)\right)}^{\alpha }\right\}+\left(\alpha -1\right)\overset{n_{1}}{\underset{i=1}{\sum }}\log\left(A\left(y_{i}\right)\right)\\ +\overset{n_{1}}{\underset{i=1}{\sum }}\left(1+r_{i}\right)\left\{1-{\left(A\left(y_{i}\right)\right)}^{\alpha }\right\}+\left(\alpha -1\right)\overset{n_{1}+n_{2}}{\underset{i=n_{1}+1}{\sum }}\text{log}\left\{B\left(y_{i}\right)\right\}+\overset{n_{1}+n_{2}}{\underset{i=n_{1}+1}{\sum }}\left(1+r_{i}\right)\left\{1-{\left(B\left(y_{i}\right)\right)}^{\alpha }\right\}. \end{array}$$

The article "Parameter Estimation in Step Stress Partially Accelerated Life Testing under Different Types of Censored Data" was published in 2022. Journal: Comput Intell Neurosci.

### 4.1. Point Estimates

Now, by differentiating (25) partially with respect to *α*, *θ*and*β*, the following equations are obtained:

(23) $$\begin{array}{c} \frac{\partial l}{\partial \alpha }=\frac{n_{1}+n_{2}}{\alpha }-n_{2}r{\left\{B\left(T_{0}\right)\right\}}^{\alpha }\text{log}\left\{B\left(T_{0}\right)\right\}+\overset{n_{1}}{\underset{i=1}{\sum }}\log\left(A\left(y_{i}\right)\right)-\overset{n_{1}}{\underset{i=1}{\sum }}\left(1+r_{i}\right){\left(A\left(y_{i}\right)\right)}^{\alpha }\log\left(A\left(y_{i}\right)\right)+\overset{n_{1}+n_{2}}{\underset{i=n_{1}+1}{\sum }}\text{log}\left\{B\left(y_{i}\right)\right\}-\overset{n_{1}+n_{2}}{\underset{i=n_{1}+1}{\sum }}\left(1+r_{i}\right){\left\{B\left(y_{i}\right)\right\}}^{\alpha }\text{log}\left\{B\left(y_{i}\right)\right\}=0, \end{array}$$

(24) $$\begin{array}{c} \frac{\partial l}{\partial \theta }=\frac{n_{1}+n_{2}}{\theta }-n_{2}r\alpha \left(\tau +\beta \left(T_{0}-\tau \right)\right){\left\{B\left(T_{0}\right)\right\}}^{\alpha -1}+\left(\alpha -1\right)\overset{n_{1}}{\underset{i=1}{\sum }}\frac{y_{i}}{\left(A\left(y_{i}\right)\right)}-\alpha \overset{n_{1}}{\underset{i=1}{\sum }}\left(1+r_{i}\right){\left(A\left(y_{i}\right)\right)}^{\alpha -1}+\overset{n_{1}+n_{2}}{\underset{i=n_{1}+1}{\sum }}\frac{B\left(y_{i}\right)-1}{\theta \left\{B\left(y_{i}\right)\right\}}-\alpha \overset{n_{1}+n_{2}}{\underset{i=n_{1}+1}{\sum }}\left(1+r_{i}\right)\frac{B\left(y_{i}\right)-1}{\theta }{\left\{B\left(y_{i}\right)\right\}}^{\alpha -1}=0, \end{array}$$

(25) $$\begin{array}{c} \frac{\partial l}{\partial \beta }=\frac{n_{2}}{\beta }-n_{2}r\theta \left(T_{0}-\tau \right){\left\{B\left(T_{0}\right)\right\}}^{\alpha -1}+\left(\alpha -1\right)\theta \overset{n_{1}+n_{2}}{\underset{i=n_{1}+1}{\sum }}\frac{\left(y_{i}-\tau \right)}{\left\{B\left(y_{i}\right)\right\}}-\alpha \theta \overset{n_{1}+n_{2}}{\underset{i=n_{1}+1}{\sum }}\left(1+r_{i}\right)\left(y_{i}-\tau \right){\left\{B\left(y_{i}\right)\right\}}^{\alpha -1}=0. \end{array}$$

The MLEs $\left(\hat{\alpha },\hat{\theta },\hat{\beta }\;\right)$ of model parameters (*α*, *θ*, *β*) under type I-PHCS can be obtained by solving equations (26)–(28) simultaneously. Unfortunately, again the system of equations (26)–(28) is nonlinear; therefore, no closed-form solution can be obtained analytically. Again, the optim () function of the R statistical software/language is implemented to solve nonlinear equations.

The article "Parameter Estimation in Step Stress Partially Accelerated Life Testing under Different Types of Censored Data" was published in 2022. Journal: Comput Intell Neurosci.

### 4.2. Interval Estimates

The same approach outlined in Subsection 3.2 can be used to produce ACIs. The entries in the Fisher information matrix are as follows:

(26) $$\begin{array}{c} \frac{\partial^{2}l}{\partial \alpha^{2}}=-\frac{n_{1}+n_{2}}{\alpha^{2}}-n_{2}r{\left\{B\left(T_{0}\right)\right\}}^{\alpha }{\left[\text{log}\left\{B\left(T_{0}\right)\right\}\right]}^{2}-\overset{n_{1}}{\underset{i=1}{\sum }}\left(1+r_{i}\right){\left(A\left(y_{i}\right)\right)}^{\alpha }{\left\{\log\left(A\left(y_{i}\right)\right)\right\}}^{2}-\overset{n_{1}+n_{2}}{\underset{i=n_{1}+1}{\sum }}\left(1+r_{i}\right){\left\{B\left(y_{i}\right)\right\}}^{\alpha }{\left[\text{log}\left\{B\left(y_{i}\right)\right\}\right]}^{2}\\ \frac{\partial^{2}l}{\partial \theta^{2}}=-\frac{n_{1}+n_{2}}{\theta^{2}}-n_{2}r\alpha \left(\alpha -1\right){\left(\frac{B\left(y_{i}\right)-1}{\theta }\right)}^{2}{\left\{B\left(T_{0}\right)\right\}}^{\alpha -1}-\left(\alpha -1\right)\overset{n_{1}}{\underset{i=1}{\sum }}\frac{y_{i}{}^{2}}{{\left(A\left(y_{i}\right)\right)}^{2}}-\alpha \left(\alpha -1\right)\overset{n_{1}}{\underset{i=1}{\sum }}\left(1+r_{i}\right)y_{i}{}^{2}{\left(A\left(y_{i}\right)\right)}^{\alpha -2}-\left(\alpha -1\right)\overset{n_{1}+n_{2}}{\underset{i=n_{1}+1}{\sum }}\frac{{\left(B\left(y_{i}\right)-1\right)}^{2}}{{\left\{\theta B\left(y_{i}\right)\right\}}^{2}}-\alpha \left(\alpha -1\right)\overset{n_{1}+n_{2}}{\underset{i=n_{1}+1}{\sum }}\left(1+r_{i}\right){\left(\frac{B\left(y_{i}\right)-1}{\theta }\right)}^{2}{\left\{B\left(y_{i}\right)\right\}}^{\alpha -2}\\ \frac{\partial^{2}l}{\partial \beta^{2}}=-\frac{n_{2}}{\beta^{2}}-n_{2}r\alpha \left(\alpha -1\right)\theta^{2}{\left(T_{0}-\tau \right)}^{2}{\left\{B\left(T_{0}\right)\right\}}^{\alpha -2}-\left(\alpha -1\right)\theta^{2}\overset{n_{1}+n_{2}}{\underset{i=n_{1}+1}{\sum }}\frac{{\left(y_{i}-\tau \right)}^{2}}{{\left\{B\left(y_{i}\right)\right\}}^{2}}-\alpha \left(\alpha -1\right)\theta^{2}\overset{n_{1}+n_{2}}{\underset{i=n_{1}+1}{\sum }}\left(1+r_{i}\right){\left(y_{i}-\tau \right)}^{2}{\left\{B\left(y_{i}\right)\right\}}^{\alpha -2}\\ \frac{\partial^{2}l}{\partial \alpha \;\partial \theta }=\frac{\partial^{2}l}{\partial \theta \;\partial \alpha }=-n_{2}r\left(\tau +\beta \left(T_{0}-\tau \right)\right){\left\{B\left(T_{0}\right)\right\}}^{\alpha -1}\left[1+\alpha \text{ log}\left\{1+\theta \left(\tau +\beta \left(T_{0}-\tau \right)\right)\right\}\right]+\overset{n_{1}}{\underset{i=1}{\sum }}\frac{y_{i}}{\left(A\left(y_{i}\right)\right)}-\overset{n_{1}}{\underset{i=1}{\sum }}\left(1+r_{i}\right)y_{i}{\left(A\left(y_{i}\right)\right)}^{\alpha -1}\left\{1+\alpha \text{ log}\left(A\left(y_{i}\right)\right)\right\}+\overset{n_{1}+n_{2}}{\underset{i=n_{1}+1}{\sum }}\frac{B\left(y_{i}\right)-1}{\theta \left\{B\left(y_{i}\right)\right\}}-\overset{n_{1}+n_{2}}{\underset{i=n_{1}+1}{\sum }}\left(1+r_{i}\right)\frac{B\left(y_{i}\right)-1}{\theta }{\left\{B\left(y_{i}\right)\right\}}^{\alpha -1}\left[1+\alpha \text{ log}\left\{B\left(y_{i}\right)\right\}\right]\\ \frac{\partial^{2}l}{\partial \alpha \;\partial \beta }=\frac{\partial^{2}l}{\partial \beta \;\partial \alpha }=-n_{2}r\theta \left(T_{0}-\tau \right){\left\{B\left(T_{0}\right)\right\}}^{\alpha -1}\left[1+\alpha \text{ log}\left\{B\left(T_{0}\right)\right\}\right]+\theta \overset{n_{1}+n_{2}}{\underset{i=n_{1}+1}{\sum }}\frac{\left(y_{i}-\tau \right)}{\left\{B\left(y_{i}\right)\right\}}-\overset{n_{1}+n_{2}}{\underset{i=n_{1}+1}{\sum }}\left(1+r_{i}\right)\left(y_{i}-\tau \right){\left\{B\left(y_{i}\right)\right\}}^{\alpha -1}\left[1+\alpha \text{ log}\left\{B\left(y_{i}\right)\right\}\right]\\ \frac{\partial^{2}l}{\partial \theta \;\partial \beta }=\frac{\partial^{2}l}{\partial \beta \;\partial \theta }=-n_{2}r\alpha \left(T_{0}-\tau \right){\left\{B\left(T_{0}\right)\right\}}^{\alpha -2}\left[1+\alpha \left(B\left(T_{0}\right)-1\right)\right]+\left(\alpha -1\right)\overset{n_{1}+n_{2}}{\underset{i=n_{1}+1}{\sum }}\frac{\left(y_{i}-\tau \right)}{{\left\{B\left(y_{i}\right)\right\}}^{2}}+\alpha \overset{n_{1}+n_{2}}{\underset{i=n_{1}+1}{\sum }}\left(1+r_{i}\right)\left(y_{i}-\tau \right){\left\{B\left(y_{i}\right)\right\}}^{\alpha -2}\left\{B\left(y_{i}\right)\right\}. \end{array}$$

The article "Parameter Estimation in Step Stress Partially Accelerated Life Testing under Different Types of Censored Data" was published in 2022. Journal: Comput Intell Neurosci.

## 5. Simulation Study

In this section, Monte Carlo simulation techniques were used to determine the unknown parameters of the distribution and AF. MLEs in type-II PCS and type-I PHCS are compared using RMSEs and RABs, whereas ACIs are compared using lengths and CPs. The simulation was run for prefixed values of *n*, *m*, *τ*, *T*_0_, and the removal scheme (*r*_1_, *r*_2_ …, *r*_*τ*_,…, *r*_*m*_). The parameters and AF are then estimated using different samples of type-II PC and type-I PHC data obtained through simulation under SSPALT. The estimation process is carried out in accordance with the following steps using numerical simulation:

Step 1: Initialize *n*, *m* *τ*and*T*_0_.
Step 2: Initialize *α*, *β*, *θ*.
Step 3: Generate type-II PC sample from NH distribution as follows:
  (i) Generate a random sample (*u*_1_, *u*_2_,…, *u*_*n*_1__) of size *n*_1_ from uniform distribution U (0, 1) with removals (*r*_1_, *r*_2_,…, *r*_*n*_1__) at stress *S*_*u*_. The failure data at stress *S*_*u*_ from the NH distribution may then be derived using the inverse CDF technique by using the following equation:
    (27) $$\begin{array}{c} y_{i}=\frac{1}{\theta }\left[{\left\{1-\log\left(1-u_{i}\right)\right\}}^{1/\alpha }-1\right]\text{if}y_{i}<\tau ,i=1,2,\ldots ,n_{1}. \end{array}$$
  (ii) Similar to step (i), the failure data at stress *S*_*a*_ from the NH distribution may then be derived by using the following equation:
  (28) $$\begin{array}{c} y_{i}=\frac{1}{\beta }\left[\frac{1}{\theta }\left\{{\left(1-\log\left(1-u_{i}\right)\right)}^{1/\alpha }-1\right\}-\tau \right]+\tau ,y_{i}>\tau ,i=1,2,\ldots ,n_{2}, \end{array}$$
  where *n*_2_=*m* − *n*_1_ and the removals are *r*_*n*_1_+1_, *r*_*n*_1_+2_,…, *r*_*m*_. At *m*^*th*^ failure *y*_*m*:*m*:*n*_, stop the test by removing all *r*_*m*_=*n* − *m* − ∑_*i*=1_^*m*−1^*r*_*i*_ survivals.
Step 4: Obtain type-I PHC data under SSPALT by repeating steps 1–3. Stop the test at *T*_0_^*∗*^=min(*y*_*m*,*m*,*n*_, *T*_0_). If *y*_*m*:*m*:*n*_ ≤ *T*_0_, stop the test at time *y*_*m*:*m*:*n*_ by removing all *r*_*m*_=*n* − *m* − ∑_*i*=1_^*m*−1^*r*_*i*_ survivals (case I). If *y*_*m*:*m*:*n*_ > *T*_0_, stop the test at time *T*_0_ by removing all *r*_*m*_=*n* − *j* − ∑_*i*=1_^*j*−1^*r*_*i*_ survivals (case II).
Step 5: Obtain the MLEs of the parameters $\Theta =\left(\hat{\alpha },\hat{\beta },\hat{\theta }\right)$ using some numerical techniques from equations (13)–(15) simultaneously for type-II PCS and from equations (26)–(28) simultaneously for type-I PHCS using the data generated in steps 1–4.
Step 6: Repeat steps 1–5 up to 10,000 times, obtain the average MLEs with their RMSEs and RABs.
Step 7: Obtain ACIs with their lengths and CPs.
Step 8: Adopt the following progressive censoring schemes for different specified sets of values of (*n*, *m*, *τ*, *T*_0_) and (*α*, *β*, *θ*) under SSPALT:
  (29) $$\begin{array}{c} \mathrm{Scheme}\;1:r_{i}=\left\{\begin{array}{cc} \left(n-m\right), & i=m,\\ 0, & \text{otherwise,} \end{array}\right.\\ \mathrm{Scheme}\;2:r_{i}=\left\{\begin{array}{cc} \left(n-1.5m+1\right), & i=m,\\ 1, & \text{otherwise,} \end{array}\right.\\ \mathrm{Scheme}\;3:r_{i}=\left\{\begin{array}{cc} \frac{\left(n-m\right)}{m}, & i=1,2,\ldots ,m\\ 0, & \text{otherwise}. \end{array}\right. \end{array}$$

Taking into account the above-mentioned algorithm, we set the initial values for (*τ*, *T*_0_) = (0.40, 0.65), (0.50, 0.80), (0.60, 1.20) and the combinations of sample sizes (*n*, *m*) = (80, 50), (80, 60), (100, 60), (100, 70), (120, 70), (120, 80). Assuming that the true values of parameters (*α*, *β*, *θ*) = (1.7, 1.3, 1.5), the MLEs of the parameters with their respective RABs and RMSEs are obtained and given in Tables 1–3 under both types of censored data. Lengths and CPs of corresponding 95% ACIs are also computed and provided in Tables 4–6.  Figure 2 depicts plots of 10000 repetitions of type-II PCS data based on SSALT. Comparative plots of RMSEs and RABs are given in Figures 3–5. Comparative plots of lengths and CPs of corresponding 95% ACIs are given in Figures 6–8.

The article "Parameter Estimation in Step Stress Partially Accelerated Life Testing under Different Types of Censored Data" was published in 2022. Journal: Comput Intell Neurosci.

From the results in Tables 1–3 and Figures 3–5, it can easily be observed that the results are consistent and the estimates are quite close to their true values for both cases of censored data. Estimates based on type-I PHCS in most of the cases are with smaller RMSEs and RABs as compared to the estimates based on type-II PCS. RMSEs and RABs are decreasing as a result of an increase in values of *n* and *m* for fixed values of (*τ*, *T*_0_) in all cases for both censoring schemes, and this is expected because the results are more accurate for large samples. The RMSEs and RABs are considerably smaller for type-I PHCS than that of type-II PCS in most of the cases. For fixed values *m*, *τ*, and *T*_0_, a decreasing pattern is observed in the values of the RMSEs and RABs with an increase in the values of *n* for type-I PHCS. The same pattern is also observed for type-II PCS but RMSEs and RABs are smaller for type-I PHCS in general for all cases. With an increase in the time of stress change *τ*, the RMSEs and RABs are decreasing for fixed values of *n*, *T*_0_, and *m*, and this is also quite obvious due to the fact that increasing the stress change time may result in more failures under normal use conditions.

For fixed values of *n*, *m*, and *τ* with an increasement in censoring time *T*_0_, RMSEs and RABs result in decreasing values for type-I PHCS, but this is not true for type-II PCS because the predetermined numbers of failures in type-II PCS, and when *T*_0_ increases, no additional failures are observed in type-II PCS. From Tables 4–6 and Figures 6–8, it is also observed that the lengths and CPs of 95% ACIs are reasonably precise for both censoring schemes in all cases but the ACIs are narrower for type-I PHCS.

As the values of *n* and *m* increase, the lengths of the ACIs decrease, and CPs are approaching 95%, and this is natural since the accuracy of the estimates depends on the size of the sample. For fixed values of *τ* and *T*_0_, with an increase in the values of *n* and *m*, the lengths of ACIs are getting narrower for all cases under the two considered censoring schemes. It is also noted that the width of ACIs for type-I PHCS is smaller than that of type-II PCS. ACIs are also getting narrower with an increasement in both stress change time *τ* and censoring time *T*_0_ for fixed values of *n* and *m* for type-I PHCS. The same pattern is true for type-II PCS, but ACIs for type-I PHCS are smaller than that of type-II PCS in general for all cases.

The article "Parameter Estimation in Step Stress Partially Accelerated Life Testing under Different Types of Censored Data" was published in 2022. Journal: Comput Intell Neurosci.

## 6. Real-Life Data Application

In this section, we will implement the models for the real data set of insulating fluid failures, which was initially reported in [64] (page 105).  Table 7 displays 19 breakdown times (in minutes) for an insulating fluid placed between two electrodes exposed to a 34 kV voltage. The goal of the experiment was to see if the time to breakdown at this voltage follows an exponential distribution as predicted by theory. If necessary, the distribution can be utilized to estimate the likelihood of fluid breakdown during real-world applications. Reference [35] investigated the data further in the context of type-II PCS, whereas [65] investigated the data in the context of adaptive type-II PCS.

We begin by verifying that the NH distribution may be utilized to examine the provided data set. The Kolmogorov–Smirnov (K–S) goodness-of-fit test is used to fit the NH distribution to real data as well as to compare the results of the NH distribution with other existing similar distributions such as the generalized exponential and Weibull generalized exponential distributions. The K–S test compares a real data set to a similar probability distribution. The test employs the K–S distance between the empirical distribution and the referenced cumulative distribution, as well as the associated *p*-values for the goodness of fit.  Table 8 shows the MLEs of unknown parameters, K–S distances, and *p*-values for all three competing distributions, including the NH, generalized exponential, and Weibull generalized exponential distributions for the considered data set. The R statistical software/language is utilized for the computation of MLEs, K–S distances, and *p*-values for each.  Figure 9 exhibits a plot of the empirical CDF versus fitted CDF, as well as a histogram of data against fitted PDF of the NH, generalized exponential, and Weibull generalized exponential distributions. From Table 8 and Figure 9, we can see that the NH distribution, when compared to the other distributions, gives a very excellent fit to the provided data set. As a result, the given data can be used as an illustration for our models.

The article "Parameter Estimation in Step Stress Partially Accelerated Life Testing under Different Types of Censored Data" was published in 2022. Journal: Comput Intell Neurosci.

Now, in SSPALT, we set the value of *τ*=7 and the total number of failures, *m*=12, which are chosen from a total of 19 (=*n*) observations, and the removal scheme, which is set to *r*_1_=*r*_2_=*r*_3_=*r*_4_=*r*_5_=*r*_6_=0, *r*_7_=*r*_8_=*r*_9_=1 at use stress level, while *r*_10_=*r*_11_=*r*_12_=0, *r*_13_=1, *r*_14_=*r*_15_=*r*_16_=0, *r*_17_=*r*_18_=*r*_19_=1 at accelerated stress level to generate the type-II PC data for illustration purpose. The generated type-II PC data is provided in Table 9. The MLEs of the parameters and their related MSEs under SSPALT with initial values of 0.497859 and 0.276878 computed for the generated type-II PC data are shown in Table 10. Similarly, we set the value of *τ*=6.5, *T*_0_=35 and the total number of failures, *m*=12, which are chosen from a total of 19 (=*n*) observations and the removal scheme, which is set to *r*_1_=*r*_2_=*r*_3_=*r*_4_=0, *r*_5_=*r*_6_=*r*_7_=1, *r*_8_=*r*_9_=*r*_10_=0 at normal stress levels and *r*_11_=0, *r*_12_=1, *r*_13_=*r*_14_=*r*_15_=0, *r*_16_=1, *r*_17_=0, *r*_18_=*r*_19_=1 at high stress levels to generate the type-I PHC data. The generated type-I PHC data is provided in Table 9. The MLEs of the parameters and their related MSEs under SSPALT with initial values of 0.497859 and 0.276878 computed for the generated type-I PHC data are shown in Table 10.

## 7. Conclusions

In this article, an SSPALT model with type-II progressively and type-I progressively hybrid censored data has been developed. Under the premise that the TRV model describes the life of the experimental units and the lifetimes of experimental units follow the NH distribution, MLEs of the unknown parameters and AF were derived. The Monte Carlo simulation study was used to compute point and interval estimates of the parameters numerically. As per the simulation results, the MLEs are fairly near to their real values and are consistent with small RMSEs and RABs for both censoring schemes. It is also noted that ACIs are relatively precise, and the predicted values for both censoring techniques fall within these ranges. As a result, it is possible to infer that the estimations are performed satisfactorily. Point estimates were compared based on their RMSEs and RABs, while interval estimates were compared based on their lengths and CPs. As a comparison between the two censoring schemes, it is found that the RMSEs and RABs for type-I PHCS are smaller than those for type-II PCS in all the sampling combinations. It is also noticed that the lengths of the ACIs of type-I PHCS are more precise than those of type-II PCS in all cases. The CPs of type-I PHCS are closer to 95% than type-I PCS. In general, it can therefore be concluded that type-I PHCS performs better than type-II PCS-based MLEs and ACs in terms of RMSEs, RABs, lengths, and CPs.

The article "Parameter Estimation in Step Stress Partially Accelerated Life Testing under Different Types of Censored Data" was published in 2022. Journal: Comput Intell Neurosci.

To demonstrate the applicability of the suggested estimation technique under SSPALT based on type-II PCS and type-I PHCS, a real-life numerical example of insulating fluid failure times is employed. As per the K–S distance and the *p*-value, the data set shows a good match for the NH distribution. To ensure that the distribution is a good fit for this data, we plotted the empirical CDF vs the fitted CDF, as well as a data histogram versus the fitted PDF of the NH distribution. In the future, the Bayesian estimation approach might be used to estimate the parameters under SSPALT for the same censoring schemes. The optimum SSPALT design can also be established in terms of the time and cost constraints on the test.

## Figures and Tables

**Figure 1:** The PDF and HRF curves with various combinations of the values of parameters.

**Figure 2:** Plots of type-II PCS data based on SSALT.

**Figure 3:** Plots of RMSEs and RABs of the estimates with *α* = 1.7, *β* = 1.3, *θ* = 1.5, and (*τ* = 0.40, *T*_0_ = 0.65): (a) type-I and type-II RMSE *α* with *t* = 0.40, *T*_0_ = 0.65; (b) type-I and type-II RAB *α* with *t* = 0.40, *T*_0_ = 0.65; (c) type-I and type-II RMSE *β* with *t* = 0.40, *T*_0_ = 0.65; (d) type-I and type-II RAB *β* with *t* = 0.40, *T*_0_ = 0.65; (e) type-I and type-II RMSE *θ* with *t* = 0.40, *T*_0_ = 0.65; and (f) type-I and type-II RAB *θ* with *t* = 0.40, *T*_0_ = 0.65.

**Figure 4:** Plots of RMSEs and RABs of the estimates with *α* = 1.7, *β* = 1.3, *θ* = 1.5, and (*τ* = 0.50, *T*_0_ = 0.80): (a) type-I and type-II RMSE *α* with *t* = 0.50, *T*_0_ = 0.80; (b) type-I and type-II RAB *α* with *t* = 0.50, *T*_0_ = 0.80; (c) type-I and type-II RMSE *β* with *t* = 0.50, *T*_0_ = 0.80; (d) type-I and type-II RAB *β* with *t* = 0.50, *T*_0_ = 0.80; (e) type-I and type-II RMSE *θ* with *t* = 0.50, *T*_0_ = 0.80; and (f) type-I and type-II RAB *θ* with *t* = 0.50, *T*_0_ = 0.80.

**Figure 5:** Plots of RMSEs and RABs of the estimates with *α* = 1.7, *β* = 1.3, *θ* = 1.5, and (*τ* = 0.60, *T*_0_ = 1.20): (a) type-I and type-II RMSE *α* with *t* = 0.60, *T*_0_ = 1.20; (b) type-I and type-II RAB *α* with *t* = 0.60, *T*_0_ = 1.20; (c) type-I and type-II RMSE *β* with *t* = 0.60, *T*_0_ = 1.20; (d) type-I and type-II RAB *β* with *t* = 0.60, *T*_0_ = 1.20; (e) type-I and type-II RMSE *θ* with *t* = 0.60, *T*_0_ = 1.20; and (f) type-I and type-II RAB *θ* with *t* = 0.60, *T*_0_ = 1.20.

The article "Parameter Estimation in Step Stress Partially Accelerated Life Testing under Different Types of Censored Data" was published in 2022. Journal: Comput Intell Neurosci.

**Figure 6:** 95% ACIs lengths and CPs of the estimates with *α* = 1.7, *β* = 1.3, *θ* = 1.5, and (*τ* = 0.40, *T*_0_ = 0.65): (a) type-I and type-II 4:95% ACIs of *α* with true values of *α* = 1.7, *β* = 1.3, *θ* = 1.5, and (*t* = 0.40, *T*_0_ = 0.65); (b) type-I and type-II 4:95% ACIs of *α* with true values of *α* = 1.7, *β* = 1.3, *θ* = 1.5, and (*t* = 0.40, *T*_0_ = 0.65); (c) type-I and type-II 4:95% ACIs of *β* with true values of *α* = 1.7, *β* = 1.3, *θ* = 1.5, and (*t* = 0.40, *T*_0_ = 0.65); (d) type-I and type-II 4:95% ACIs of *β* with true values of *α* = 1.7, *β* = 1.3, *θ* = 1.5, and (*t* = 0.40, *T*_0_ = 0.65); (e) type-I and type-II 95% ACIs of *θ* with true values of *α* = 1.7, *β* = 1.3, *θ* = 1.5, and (*t* = 0.50, *T*_0_ = 0.80); and (f) type-I and type-II 4:95% ACIs of *θ* with true values of *α* = 1.7, *β* = 1.3, *θ* = 1.5, and (*t* = 0.40, *T*_0_ = 0.65).

**Figure 7:** 95% ACIs lengths and CPs of the estimates with *α* = 1.7, *β* = 1.3, *θ* = 1.5, and (*τ* = 0.50, *T*_0_ = 0.80): (a) type-I and type-II 95% ACIs of *α* with true values of *α* = 1.7, *β* = 1.3, *θ* = 1.5, and (*t* = 0.50, *T*_0_ = 0.80); (b) type-I and type-II 5:95% ACIs of *α* with true values of *α* = 1.7, *β* = 1.3, *θ* = 1.5, and (*t* = 0.50, *T*_0_ = 0.80); (c) type-I and type-II 95% ACIs of *β* with true values of *α* = 1.7, *β* = 1.3, *θ* = 1.5, and (*t* = 0.50, *T*_0_ = 0.80); (d) type-I and type-II 5:95% ACIs of *β* with true values of *α* = 1.7, *β* = 1.3, *θ* = 1.5, and (*t* = 0.50, *T*_0_ = 0.80); (e) type-I and type-II 95% ACIs of *θ* with true values of *α* = 1.7, *β* = 1.3, *θ* = 1.5, and (*t* = 0.50, *T*_0_ = 0.80); and (f) type-I and type-II 5:95% ACIs of *θ* with true values of *α* = 1.7, *β* = 1.3, *θ* = 1.5, and (*t* = 0.50, *T*_0_ = 0.80).

**Figure 8:** 95% ACIs Lengths and CPs of the estimates with *α* = 1.7, *β* = 1.3, *θ* = 1.5, and (*τ* = 0.60, *T*_0_ = 1.20): (a) type-I and type-II 95% ACIs of *α* with true values of *α* = 1.7, *β* = 1.3, *θ* = 1.5, and (*t* = 0.60, *T*_0_ = 1.20); (b) type-I and type-II 95% ACIs of *α* with true values of *α* = 1.7, *β* = 1.3, *θ* = 1.5, and (*t* = 0.60, *T*_0_ = 1.20); (c) type-I and type-II 95% ACIs of *β* with true values of *α* = 1.7, *β* = 1.3, *θ* = 1.5, and (*t* = 0.60, *T*_0_ = 1.20); (d) type-I and type-II 95% ACIs of *β* with true values of *α* = 1.7, *β* = 1.3, *θ* = 1.5, and (*t* = 0.60, *T*_0_ = 1.20); (e) type-I and type-II 95% ACIs of *θ* with true values of *α* = 1.7, *β* = 1.3, *θ* = 1.5, and (*t* = 0.60, *T*_0_ = 1.20); and (f) type-I and type-II 95% ACIs of *θ* with true values of *α* = 1.7, *β* = 1.3, *θ* = 1.5, and (*t* = 0.60, *T*_0_ = 1.20).

The article "Parameter Estimation in Step Stress Partially Accelerated Life Testing under Different Types of Censored Data" was published in 2022. Journal: Comput Intell Neurosci.

**Figure 9:** (a) Plot of the empirical CDF versus fitted CDF and (b) histogram of data against fitted PDF.

**Table 1:** MLEs, RMSEs, and RABs with true values of *α* = 1.7, *β* = 1.3, *θ* = 1.5, and (*τ* = 0.40, *T*_0_ = 0.65).

(*n*, *m*)	CS	Type-II PCS									Type-I PHCS								
		*α*			*β*			*θ*			*α*			*β*			*θ*		
		MLE	RMSE	RAB	MLE	RMSE	RAB	MLE	RMSE	RAB	MLE	RMSE	RAB	MLE	RMSE	RAB	MLE	RMSE	RAB
(80, 50)	1	1.725	0.491	0.312	1.625	0.506	0.361	1.693	0.486	0.327	1.895	0.129	0.054	1.462	0.421	0.312	1.695	0.273	0.213
(80, 60)	1	1.73	0.459	0.301	1.542	0.516	0.358	1.658	0.447	0.319	1.797	0.106	0.086	1.189	0.311	0.257	1.78	0.268	0.213
(100, 60)	1	1.688	0.413	0.284	1.493	0.451	0.311	1.743	0.426	0.312	1.857	0.098	0.068	1.199	0.287	0.218	1.755	0.255	0.199
(100, 70)	1	1.675	0.426	0.275	1.506	0.334	0.304	1.567	0.376	0.302	1.645	0.098	0.064	1.193	0.291	0.207	1.673	0.251	0.206
(120, 70)	1	1.714	0.399	0.262	1.452	0.32	0.243	1.544	0.329	0.239	1.574	0.078	0.013	1.382	0.269	0.198	1.68	0.246	0.201
(120, 80)	1	1.618	0.381	0.227	1.482	0.285	0.217	1.606	0.309	0.213	1.493	0.018	0.004	1.318	0.252	0.193	1.681	0.229	0.184
(80, 50)	2	1.713	0.527	0.308	1.496	0.519	0.359	1.875	0.552	0.387	1.787	0.114	0.074	1.498	0.337	0.279	1.738	0.264	0.215
(80, 60)	2	1.694	0.446	0.299	1.505	0.518	0.354	1.723	0.464	0.326	1.513	0.11	0.072	1.136	0.323	0.248	1.716	0.263	0.211
(100, 60)	2	1.73	0.458	0.291	1.439	0.51	0.317	1.705	0.426	0.297	1.79	0.099	0.071	1.21	0.297	0.226	1.669	0.254	0.207
(100, 70)	2	1.756	0.433	0.287	1.407	0.451	0.254	1.599	0.367	0.313	1.752	0.028	0.009	1.471	0.291	0.216	1.692	0.244	0.204
(120, 70)	2	1.619	0.404	0.253	1.535	0.384	0.254	1.831	0.362	0.274	1.71	0.018	0.005	1.509	0.278	0.211	1.784	0.232	0.199
(120, 80)	2	1.66	0.376	0.211	1.503	0.321	0.241	1.581	0.35	0.264	1.683	0.011	0.004	1.598	0.227	0.183	1.663	0.215	0.186
(80, 50)	3	1.716	0.489	0.303	1.598	0.447	0.384	1.802	0.527	0.358	1.754	0.128	0.078	1.486	0.404	0.294	1.727	0.259	0.207
(80, 60)	3	1.758	0.424	0.296	1.569	0.412	0.366	1.806	0.478	0.352	1.448	0.119	0.091	1.057	0.309	0.255	1.754	0.254	0.209
(100, 60)	3	1.691	0.422	0.293	1.554	0.387	0.331	1.756	0.368	0.328	1.787	0.097	0.069	1.264	0.273	0.231	1.759	0.253	0.209
(100, 70)	3	1.727	0.42	0.283	1.497	0.405	0.295	1.696	0.356	0.278	1.729	0.037	0.013	1.129	0.266	0.203	1.668	0.233	0.194
(120, 70)	3	1.621	0.398	0.279	1.513	0.388	0.263	1.761	0.395	0.258	1.663	0.037	0.009	1.269	0.266	0.208	1.724	0.228	0.175
(120, 80)	3	1.67	0.399	0.226	1.524	0.301	0.225	1.606	0.378	0.257	1.807	0.017	0.005	1.473	0.248	0.189	1.689	0.215	0.172

**Table 2:** MLEs, RMSEs, and RABs with true values of *α* = 1.7, *β* = 1.3, *θ* = 1.5, and (*τ* = 0.50, *T*_0_ = 0.80).

(*n*, *m*)	CS	Type-II PCS									Type-I PHCS								
		*α*			*β*			*θ*			*α*			*β*			*θ*		
		MLE	RMSE	RAB	MLE	RMSE	RAB	MLE	RMSE	RAB	MLE	RMSE	RAB	MLE	RMSE	RAB	MLE	RMSE	RAB
(80, 50)	1	1.713	0.525	0.436	1.498	0.411	0.341	1.678	0.529	0.439	1.885	0.58	0.481	1.486	0.56	0.465	1.687	0.272	0.226
(80, 60)	1	1.725	0.48	0.398	1.602	0.37	0.307	1.598	0.434	0.36	1.875	0.415	0.344	1.519	0.335	0.278	1.687	0.26	0.216
(100, 60)	1	1.692	0.462	0.383	1.62	0.33	0.274	1.771	0.406	0.337	1.578	0.33	0.274	1.497	0.33	0.274	1.763	0.253	0.21
(100, 70)	1	1.62	0.454	0.366	1.603	0.309	0.256	1.554	0.406	0.337	1.799	0.29	0.241	1.469	0.305	0.253	1.737	0.243	0.202
(120, 70)	1	1.658	0.434	0.356	1.496	0.285	0.237	1.68	0.397	0.33	1.641	0.265	0.22	1.436	0.301	0.25	1.738	0.232	0.193
(120, 80)	1	1.762	0.424	0.348	1.593	0.285	0.237	1.579	0.378	0.314	1.694	0.027	0.022	1.522	0.274	0.227	1.681	0.212	0.176
(80, 50)	2	1.717	0.534	0.443	1.583	0.373	0.31	1.872	0.449	0.373	1.774	0.618	0.513	1.493	0.629	0.522	1.754	0.336	0.279
(80, 60)	2	1.729	0.479	0.398	1.56	0.332	0.276	1.643	0.435	0.361	1.773	0.469	0.389	1.344	0.332	0.276	1.688	0.277	0.23
(100, 60)	2	1.612	0.421	0.349	1.492	0.315	0.261	1.971	0.39	0.324	1.685	0.435	0.361	1.626	0.331	0.275	1.734	0.257	0.213
(100, 70)	2	1.759	0.417	0.346	1.481	0.315	0.261	1.534	0.384	0.319	1.603	0.237	0.197	1.511	0.301	0.25	1.721	0.253	0.21
(120, 70)	2	1.687	0.397	0.33	1.575	0.283	0.235	1.714	0.381	0.316	1.591	0.15	0.125	1.614	0.266	0.221	1.709	0.227	0.188
(120, 80)	2	1.654	0.356	0.295	1.597	0.236	0.196	1.62	0.303	0.251	1.536	0.149	0.124	1.526	0.257	0.213	1.725	0.213	0.177
(80, 50)	3	1.738	0.473	0.393	1.605	0.407	0.338	1.502	0.465	0.386	1.851	0.589	0.489	1.529	0.425	0.353	1.718	0.256	0.212
(80, 60)	3	1.712	0.449	0.373	1.401	0.375	0.311	1.892	0.44	0.365	1.557	0.475	0.394	1.603	0.304	0.252	1.717	0.253	0.21
(100, 60)	3	1.755	0.446	0.37	1.369	0.327	0.271	1.832	0.402	0.334	1.879	0.344	0.286	1.498	0.303	0.251	1.744	0.251	0.208
(100, 70)	3	1.692	0.409	0.339	1.604	0.319	0.265	1.498	0.396	0.329	1.766	0.267	0.222	1.257	0.287	0.238	1.659	0.235	0.195
(120, 70)	3	1.661	0.378	0.314	1.538	0.31	0.257	1.822	0.379	0.315	1.627	0.259	0.215	1.509	0.278	0.231	1.813	0.205	0.17
(120, 80)	3	1.619	0.356	0.295	1.542	0.305	0.253	1.534	0.292	0.242	1.677	0.105	0.087	1.309	0.273	0.227	1.712	0.202	0.168

The article "Parameter Estimation in Step Stress Partially Accelerated Life Testing under Different Types of Censored Data" was published in 2022. Journal: Comput Intell Neurosci.

**Table 3:** MLEs, RMSEs, and RABs with true values of *α* = 1.7, *β* = 1.3, *θ* = 1.5, and (*τ* = 0.60, *T*_0_ = 1.20).

(*n*, *m*)	CS	Type-II PCS									Type-I PHCS								
		*α*			*β*			*θ*			*α*			*β*			*θ*		
		MLE	RMSE	RAB	MLE	RMSE	RAB	MLE	RMSE	RAB	MLE	RMSE	RAB	MLE	RMSE	RAB	MLE	RMSE	RAB
(80, 50)	1	1.73	0.528	0.438	1.497	0.411	0.341	1.761	0.43	0.357	1.536	0.376	0.312	1.261	0.464	0.385	1.667	0.274	0.227
(80, 60)	1	1.714	0.456	0.378	1.402	0.347	0.288	1.581	0.429	0.356	1.811	0.285	0.237	1.261	0.399	0.331	1.742	0.265	0.22
(100, 60)	1	1.76	0.435	0.361	1.569	0.339	0.281	1.843	0.363	0.301	1.528	0.194	0.161	1.484	0.295	0.245	1.753	0.262	0.217
(100, 70)	1	1.689	0.397	0.33	1.582	0.314	0.261	1.922	0.348	0.289	1.605	0.165	0.137	1.337	0.278	0.231	1.731	0.245	0.203
(120, 70)	1	1.621	0.377	0.313	1.505	0.309	0.256	1.842	0.346	0.287	1.753	0.133	0.11	1.408	0.258	0.214	1.69	0.219	0.182
(120, 80)	1	1.668	0.375	0.311	1.535	0.225	0.187	1.777	0.32	0.266	1.698	0.057	0.047	1.516	0.234	0.194	1.714	0.216	0.179
(80, 50)	2	1.722	0.51	0.423	1.463	0.473	0.393	1.99	0.446	0.371	1.561	0.517	0.429	1.256	0.438	0.364	1.701	0.28	0.232
(80, 60)	2	1.74	0.436	0.362	1.452	0.401	0.333	1.842	0.443	0.368	1.78	0.353	0.293	1.324	0.307	0.255	1.73	0.266	0.221
(100, 60)	2	1.684	0.39	0.324	1.413	0.295	0.245	1.664	0.388	0.322	1.542	0.247	0.205	1.306	0.306	0.254	1.809	0.226	0.188
(100, 70)	2	1.62	0.389	0.323	1.437	0.289	0.24	1.694	0.365	0.303	1.898	0.207	0.172	1.2	0.281	0.233	1.715	0.223	0.185
(120, 70)	2	1.66	0.389	0.323	1.478	0.287	0.238	1.715	0.361	0.305	1.946	0.191	0.159	1.523	0.254	0.211	1.684	0.213	0.177
(120, 80)	2	1.755	0.377	0.313	1.53	0.237	0.197	1.898	0.334	0.277	1.963	0.184	0.153	1.409	0.246	0.204	1.723	0.21	0.174
(80, 50)	3	1.712	0.482	0.4	1.609	0.382	0.317	1.782	0.395	0.328	1.598	0.642	0.533	1.359	0.541	0.449	1.694	0.284	0.236
(80, 60)	3	1.734	0.463	0.384	1.398	0.332	0.276	1.658	0.384	0.319	1.518	0.398	0.33	1.372	0.303	0.251	1.744	0.268	0.222
(100, 60)	3	1.688	0.434	0.36	1.581	0.321	0.266	1.772	0.333	0.276	1.725	0.296	0.246	1.265	0.289	0.24	1.717	0.264	0.219
(100, 70)	3	1.615	0.415	0.344	1.515	0.274	0.227	1.924	0.328	0.272	1.683	0.258	0.214	1.405	0.28	0.232	1.693	0.237	0.197
(120, 70)	3	1.756	0.381	0.316	1.513	0.235	0.195	1.694	0.326	0.271	1.701	0.147	0.122	1.393	0.244	0.203	1.775	0.233	0.193
(120, 80)	3	1.66	0.374	0.31	1.395	0.234	0.194	1.84	0.322	0.267	1.652	0.139	0.115	1.452	0.222	0.184	1.717	0.181	0.15

**Table 4:** Lengths and CPs of 95% ACIs with *α* = 1.7, *β* = 1.3, *θ* = 1.5, and (*τ* = 0.40, *T*_0_ = 0.65).

(*n*, *m*)	CS	Type-II PCS						Type-I PHCS					
		*α*		*β*		*θ*		*α*		*β*		*θ*	
		Length	CP	Length	CP	Length	CP	Length	CP	Length	CP	Length	CP
(80, 50)	1	1.924	94.87	1.044	95.06	1.906	94.91	0.506	94.48	0.694	95.01	1.07	94.61
(80, 60)	1	1.8	94.96	0.798	94.57	1.752	94.67	0.416	94.39	0.38	94.33	1.05	94.26
(100, 60)	1	1.67	94.58	0.558	94.85	1.67	94.99	0.384	94.07	0.332	94.22	1.01	95.01
(100, 70)	1	1.618	94.93	0.438	94.67	1.474	94.16	0.306	94.86	0.286	94.86	0.984	94.37
(120, 70)	1	1.564	95.13	0.402	94.64	1.29	94.71	0.235	94.61	0.284	94.39	0.964	94.33
(120, 80)	1	1.494	94.79	0.318	94.28	1.212	95.04	0.172	94.65	0.248	94.69	0.862	94.86
(80, 50)	2	2.066	95.04	1.056	95.04	2.164	94.61	0.446	94.24	0.446	94.93	1.034	94.76
(80, 60)	2	1.796	94.92	1.052	93.99	1.818	94.86	0.432	95.06	0.408	94.56	1.02	94.71
(100, 60)	2	1.748	95.08	1.02	95.03	1.67	94.93	0.11	95.04	0.346	94.14	0.956	94.63
(100, 70)	2	1.698	95.07	0.798	94.96	1.438	94.56	0.078	94.2	0.332	94.61	0.91	94.65
(120, 70)	2	1.584	94.87	0.578	94.49	1.42	94.78	0.07	94.82	0.302	94.07	0.842	94.14
(120, 80)	2	1.474	94.69	0.404	94.78	1.372	94.44	0.044	94.37	0.202	94.67	0.784	94.56
(80, 50)	3	1.916	94.94	2.584	94.89	2.066	94.54	0.502	94.93	0.64	94.29	1.016	95.04
(80, 60)	3	1.662	94.97	0.784	94.73	1.842	94.65	0.466	94.91	0.374	94.46	0.996	94.18
(100, 60)	3	1.654	95.02	0.642	95.01	1.63	94.52	0.188	94.97	0.292	94.26	0.992	94.69
(100, 70)	3	1.646	94.63	0.59	94.63	1.56	94.84	0.146	94.26	0.278	94.41	0.914	94.24
(120, 70)	3	1.564	95.12	0.398	94.71	1.396	94.39	0.146	94.59	0.278	94.44	0.894	94.48
(120, 80)	3	1.56	94.76	0.356	94.37	1.352	94.89	0.066	94.14	0.242	94.71	0.842	94.11

The article "Parameter Estimation in Step Stress Partially Accelerated Life Testing under Different Types of Censored Data" was published in 2022. Journal: Comput Intell Neurosci.

**Table 5:** Lengths and CPs of 95% ACIs with *α* = 1.7, *β* = 1.3, *θ* = 1.5, and (*τ* = 0.50, *T*_0_ = 0.80).

(*n*, *m*)	CS	Type-II PCS						Type-I PHCS					
		*α*		*β*		*θ*		*α*		*β*		*θ*	
		Length	CP	Length	CP	Length	CP	Length	CP	Length	CP	Length	CP
(80, 50)	1	2.058	94.59	0.662	93.99	2.074	94.18	2.274	94.87	1.23	94.37	1.066	93.99
(80, 60)	1	1.882	95.17	0.536	94.92	1.702	94.04	1.626	94.4	0.44	95.17	1.02	93.91
(100, 60)	1	1.812	93.93	0.426	94.87	1.592	93.93	1.294	94.43	0.426	94.9	0.992	94.7
(100, 70)	1	1.702	94.65	0.374	94.32	1.592	94.13	1.136	95.09	0.364	94.29	0.952	94.37
(120, 70)	1	1.702	93.96	0.318	94.57	1.556	95.09	1.038	95.06	0.356	93.96	0.91	94.73
(120, 80)	1	1.702	94.02	0.318	94.84	1.482	94.81	0.106	95.17	0.294	94.26	0.832	94.29
(80, 50)	2	2.094	94.4	0.546	94.37	1.76	93.96	2.422	95.01	1.55	94.1	1.318	94.15
(80, 60)	2	1.878	94.26	0.432	95.14	1.706	94.92	1.838	94.15	0.432	94.18	1.086	94.57
(100, 60)	2	1.65	94.79	0.388	95.09	1.528	94.84	1.706	94.95	0.43	94.57	1.008	94.18
(100, 70)	2	1.634	94.54	0.388	94.62	1.506	94.46	0.93	94.46	0.356	94.73	0.992	94.62
(120, 70)	2	1.556	93.88	0.314	95.17	1.494	93.88	0.588	94.37	0.278	95.01	0.89	94.81
(120, 80)	2	1.396	94.29	0.218	94.02	1.188	94.65	0.584	94.9	0.258	94.87	0.834	95.09
(80, 50)	3	1.854	94.81	0.65	94.54	1.822	95.2	2.308	94.51	0.708	93.91	1.004	95.03
(80, 60)	3	1.76	94.35	0.552	95.12	1.724	94.87	1.862	94.24	0.362	94.21	0.992	94.48
(100, 60)	3	1.748	94.46	0.42	95.01	1.576	95.17	1.348	93.88	0.36	94.4	0.984	94.02
(100, 70)	3	1.604	94.87	0.398	94.7	1.552	94.24	1.046	94.54	0.322	94.07	0.922	94.32
(120, 70)	3	1.482	94.51	0.376	94.26	1.486	94.54	1.016	94.32	0.302	93.99	0.804	94.95
(120, 80)	3	1.396	94.37	0.364	94.98	1.144	95.06	0.412	94.62	0.292	94.24	0.792	94.07

The article "Parameter Estimation in Step Stress Partially Accelerated Life Testing under Different Types of Censored Data" was published in 2022. Journal: Comput Intell Neurosci.

**Table 6:** Lengths and CPs of 95% ACIs with *α* = 1.7, *β* = 1.3, *θ* = 1.5, and (*τ* = 0.60, *T*_0_ = 1.20).

(*n*, *m*)	CS	Type-II PCS						Type-I PHCS					
		*α*		*β*		*θ*		*α*		*β*		*θ*	
		Length	CP	Length	CP	Length	CP	Length	CP	Length	CP	Length	CP
(80, 50)	1	2.07	94.57	0.662	94.54	1.686	94.87	1.474	93.79	0.844	94.73	1.074	94.79
(80, 60)	1	1.788	94.9	0.472	93.82	1.682	94.98	1.118	95.04	0.624	93.79	1.038	94.26
(100, 60)	1	1.706	94.96	0.45	94.9	1.422	95.09	0.76	94.65	0.342	94.32	1.028	95.07
(100, 70)	1	1.556	94.87	0.386	94.21	1.364	93.87	0.646	94.87	0.302	94.93	0.96	94.57
(120, 70)	1	1.478	94.15	0.374	94.29	1.356	94.01	0.522	94.15	0.26	94.1	0.858	93.85
(120, 80)	1	1.47	93.82	0.198	94.01	1.254	94.29	0.224	93.85	0.214	94.9	0.846	94.98
(80, 50)	2	2.002	94.54	0.878	93.87	1.748	93.79	2.026	94.21	0.752	95.09	1.098	94.62
(80, 60)	2	1.71	94.51	0.63	93.79	1.736	94.51	1.384	94.84	0.37	93.98	1.042	94.93
(100, 60)	2	1.528	94.93	0.342	94.35	1.52	94.59	0.968	94.51	0.368	94.87	0.886	94.65
(100, 70)	2	1.524	94.23	0.328	94.93	1.43	93.96	0.812	95.09	0.31	95.04	0.874	94.01
(120, 70)	2	1.524	94.82	0.322	95.09	1.416	94.35	0.748	93.96	0.252	95.12	0.834	94.37
(120, 80)	2	1.478	93.87	0.22	94.84	1.31	94.71	0.722	94.07	0.238	94.84	0.824	95.09
(80, 50)	3	1.89	94.01	0.572	94.15	1.548	93.85	2.516	94.23	1.148	94.96	1.114	94.71
(80, 60)	3	1.814	94.26	0.432	94.68	1.506	93.98	1.56	94.71	0.36	94.62	1.05	94.04
(100, 60)	3	1.702	94.18	0.404	94.23	1.306	94.04	1.16	94.1	0.328	94.26	1.034	94.54
(100, 70)	3	1.626	94.59	0.294	94.1	1.286	94.79	1.012	94.73	0.308	94.4	0.93	93.87
(120, 70)	3	1.494	94.21	0.216	94.76	1.278	94.37	0.576	93.93	0.234	94.21	0.914	94.21
(120, 80)	3	1.466	94.73	0.214	94.65	1.262	94.68	0.544	95.12	0.194	94.82	0.71	94.84

**Table 7:** Insulating fluid data.

0.19	0.78	0.96	1.31	2.78	3.16	4.15	4.67	4.85	6.50
7.35	8.01	8.27	12.06	31.75	32.52	33.91	36.71	72.89	

**Table 8:** MLEs, K–S distances, and *p*-values based on complete insulating fluid data.

Distribution	Alpha	Beta	Theta	K–S test	*p*-value
NH distribution	0.497859	0.276878	—	0.14238	0.7855
Weibull generalized exponential	15.121028	0.002218	0.785	0.20329	0.3625
Generalized exponential	0.803419	0.102165	—	0.22958	0.2309

**Table 9:** The generated type-II PC and type-I PHC data sets.

Type-II PC data	Normal stress: 0.19, 0.78, 0.96, 1.31, 2.78, 3.16, 6.50
	Accelerated stress: 7.35, 8.01, 12.06, 31.75, 32.52

Type-I PHC data	Normal stress: 0.19, 0.78, 0.96, 1.31, 4.67, 4.85, 6.50
	Accelerated stress: 7.35, 8.27, 12.06, 31.75, 33.91

**Table 10:** MLEs with their related MSEs under SSPALT.

Censoring	$\hat{\alpha }$		$\hat{\beta }$		$\hat{\theta }$	
	MLE	MSE	MLE	MSE	MLE	MSE
Type-II PCS	0.895165	0.00234	0.358743	0.00198	1.201932	0.000365
Type-II PHCS	0.942767	0.000823	0.462885	0.000519	1.266381	0.000173

The article "Parameter Estimation in Step Stress Partially Accelerated Life Testing under Different Types of Censored Data" was published in 2022. Journal: Comput Intell Neurosci.

## Data Availability

All data used to support the findings are available in the paper.
